The article "Investigating the Effect of Keyboard Distance on the Posture and 3D Moments of Wrist and Elbow Joints among Males Using OpenSim" was published in 2022. Journal: Appl Bionics Biomech.

# Investigating the Effect of Keyboard Distance on the Posture and 3D Moments of Wrist and Elbow Joints among Males Using OpenSim

**DOI:** 10.1155/2022/5751488

**Published:** 2022-05-05

**Authors:** Milad Gholami, Alireza Choobineh, Mohammad Abdoli-Eramaki, Azizallah Dehghan, Mohammad Taghi Karimi

**Affiliations:** ^1^Department of Ergonomics, Student Research Committee, Shiraz University of Medical Sciences, Shiraz, Iran; ^2^Research Center for Health Sciences, Institute of Health, Shiraz University of Medical Sciences, Shiraz, Iran; ^3^School of Occupational and Public Health, Ryerson University, Toronto, Canada; ^4^Noncommunicable Diseases Research Center, Fasa University of Medical Sciences, Fasa, Iran; ^5^School of Rehabilitation Sciences, Shiraz University of Medical Sciences, Shiraz, Iran

## Abstract

Musculoskeletal disorders (MSDs) of the upper extremities and computer use are common in modern societies, and both show a growing trend. This study was conducted to determine the posture and 3D moments of wrist and elbow joints at different keyboard distances on a desk. Twelve healthy right-handed male volunteers attended the motion analysis laboratory. A keyboard was placed at three different distances from the participants' bodies while performing a standard computer task. The workstation was adjusted according to ANSI/HFES-100-2007 standard for each participant to maintain a comfortable ergonomic posture for controlling confounding variables. Qualisys motion capture system, OpenSim (Ver. 4.1), and visual analog scale were used to collect and analyze the data. The highest levels of wrist flexion and radial deviation as well as elbow flexion and pronation were observed when the keyboard was at the edge of the desk. When the keyboard was 8 cm away from the edge of the desk, the right wrist flexion and radial deviation decreased 83% and 89%, respectively. In the left wrist, flexion and radial deviation decreased 94%. With increasing the distance of the keyboard from the edge of the desk, the right elbow flexion, pronation, and left elbow flexion decreased, 95%, 76%, and 85%, respectively. No significant difference was found for the left elbow pronation, wrist, and elbow joint moments, in the studied keyboard distances. However, a cut-off point has to be specified because large keyboard distances cause high extension and flexion of the limbs. The keyboard position relative to the body is an important parameter in computer work and has a significant impact on the posture of the upper extremities. A keyboard should be located at a distance that allows the upper extremities to remain in a neutral position so that the risk of MSDs is reduced.

## 1. Introduction

Musculoskeletal disorders (MSDs) of the upper extremities and computer use are common in modern societies, and both show a growing trend. Many studies have discussed a possible relationship between computer work and musculoskeletal problems in the upper extremities [1–3]. Workstation factors that may increase the risk of upper extremity symptoms and disorders include lack of armrests and inappropriate keyboard location [4, 5]. These problems usually occur when operators have poor postures and have to work in this situation for a long time [6]. Existing guidelines for computer workstation designs are based on anthropometric measurements, while biomechanics and computer user behavior patterns are also important variables in developing musculoskeletal disorders [7].

The article "Investigating the Effect of Keyboard Distance on the Posture and 3D Moments of Wrist and Elbow Joints among Males Using OpenSim" was published in 2022. Journal: Appl Bionics Biomech.

Evidence suggests that workstation parameters are associated with the development of MSDs [8, 9]. Marcus et al. showed the association of various workstation and postural factors with musculoskeletal symptoms in a large longitudinal epidemiological study. Most recommendations highlight modification of the body posture as the mainstay of risk reduction in computer users [10]. Sauter et al., for example, reported that arm discomfort increased with keyboard height above elbow level [11]. Risk factors linked to computer use include physical ergonomic factors such as desk, chair, monitor height, postures, and the use of input devices such as computer keyboard and mouse [12]. Upper extremity musculoskeletal disorders (UEMSDs) are associated with the use of keyboard and visual display unit (VDU) [13]. The prevalence of these disorders among Iranian office workers is 56.6% in the neck, 38.2% in the shoulder, 15% in the elbow, and 46.7% in the wrist [14].

Computer workstation design is the main goal in ergonomics for preventing or minimizing work-related MSDs [15]. An essential factor in workstations that increases the risk of shoulder and hand disorders is the placement of the keyboard and the lack of forearm support [10, 16]. The keyboard location and its distance from the edge of the desk affect the posture and moments of hands, wrists, elbows, and arms [17]. Repetitive motions and awkward postures in the computer keyboard typing are risk factors for computer-related MSDs [18]. The wrist flexion-extension and ulnar-radial deviation, as well as elbow rotation (supination-pronation), are important factors in causing MSDs, so that higher values of these variables increase the risk of MSDs. Additionally, high values of joint moment are directly related to MSDs and affect the incidence of these disorders. If these parameters are not considered in the design and placement of keyboards, the risk of upper extremity injuries increases [11].

The article "Investigating the Effect of Keyboard Distance on the Posture and 3D Moments of Wrist and Elbow Joints among Males Using OpenSim" was published in 2022. Journal: Appl Bionics Biomech.

However, very few studies have been done on the effect of the horizontal distance of the keyboard in the design of computer workstations. There are limited findings on the impact of these parameters and their relationship with MSDs in the upper extremities [19]. Many studies have been conducted on variables such as slope, shape, and palm rest of the keyboard, and few studies indirectly have measured posture and muscle forces to recognize the effect of the horizontal distance of the keyboard from the edge of the desk on the posture and muscle forces [12, 19, 20].

Common pen-paper evaluation methods such as Rapid Upper Limb Assessment (RULA), Loading Postural Upper Body Assessment (LUBA), and Ovako Working Posture Assessment System (OWAS), which are widely used in the ergonomic evaluation. Ergonomics methods (instrumental, observational, and self-report) assess posture parameters, such as proximity of the joint end stops, implied loads, time, and repetition. However, these methods do not take into account the behavior of biological tissues which are yet largely at the origin of the discomfort feeling [21]. Also, an electromyography recording (EMG) can show when a muscle is active, but examining an EMG recording does not determine which body motions are caused by muscle activity [22]. Dynamic simulations of the musculoskeletal system are becoming a viable approach for specifying how the musculoskeletal system's elements interact to the movement process. A dynamic simulation of movement that integrates models describing the anatomy and physiology of the elements of the neuromusculoskeletal system and the mechanics of multijoint movement provides such a framework. Muscle-driven dynamic simulations complement experimental approaches by providing estimates of important variables, such as muscle and joint forces, which are difficult to measure experimentally [23]. To quantify the elements that affect the MSDs and prevent the potential disorders, a three-dimensional muscle-actuated simulator with the ability to accurately reproduce the individual dynamic movement is beneficial [24]. OpenSim has been widely used for modelling the musculoskeletal system while visualizing the motion. It is able to quantify joint position, muscle forces, and moments using inverse kinematics and dynamics [25].

Studying and controlling MSDs through software methods such as MATLAB, CAD, and Bond graph developed in neuromuscular biomechanics can significantly reduce the costs compared to treatment and rehabilitation approaches [26, 27]. Many studies have used computers and input devices, such as keyboard and keyboard tray, while the use of keyboard tray is not yet common in Iran. Musculoskeletal models allow the estimation of muscle function during complex tasks. Therefore, using OpenSim as a modern and objective biomechanical evaluation method, this study was aimed at determining the effect of keyboard distance on the posture and 3D moments of wrist and elbow joints. It is believed that the findings can be used in product design and the development of standards for computer use.

The article "Investigating the Effect of Keyboard Distance on the Posture and 3D Moments of Wrist and Elbow Joints among Males Using OpenSim" was published in 2022. Journal: Appl Bionics Biomech.

## 2. Materials and Methods

An experimental study was conducted on twelve randomly selected healthy males aged from 25 to 30 years with no history of any MSDs. To prevent the probable dominant hand confounding effect, all participants were selected among right-handed individuals. Individuals who entered the study were familiar with computer use, and their mean (SD) of typing speed was 45.37 (11.67) words per minute (ranged from 25 to 87 words per minute).

Ethics approval was obtained through the Shiraz University of Medical Sciences Ethics Committee (IR.SUMS.REHAB.REC.1399.021), and all participants provided fully informed consent for participation in this study, and all methods were carried out in accordance with Helsinki approved guidelines and regulations.

The inclusion criteria were having a height of 165-185 cm, working with computer for 3-4 hours a day, and being right-handed. Exclusion criteria included the history of any MSDs in any body region. This study used Qualisys motion capture system, OpenSim software (version 4.1), and VAS to collect and analyze data.

### 2.1. Qualisys Motion Capture System

Qualisys motion analysis system was calibrated and used with eight high-speed cameras at a frequency of 120 Hz. The magnitude error of the motion analysis system for each camera was less than 1 millimeter. The data obtained in this section was first defined based on anatomical points (labeling) and was stored in C3D format and then converted into TRC format using Mokka software (version 0.6) to be compatible with the OpenSim software for further biomechanical analysis.

### 2.2. OpenSim

OpenSim software calculated the joint kinematics and kinetics using inverse kinematics and inverse dynamics. Both hands' wrist flexion-extension, ulnar-radial deviation, elbow flexion-extension, and supination-pronation movements were evaluated using OpenSim. After entering the motion analysis data into OpenSim and using the Rajagopal model to perform scaling (Figure 1), the angles of the joints and their range of motion (ROM) were calculated. In this section, the wrist and elbow joints were selected to calculate their angles and moments separately. In this study, there was no external force and only the upper limbs force was considered, which was added to model by the OpenSim software in the scaling stage and based on the center of mass in each upper limb section. To calculate the moment of the wrists and elbow, OpenSim Inverse Dynamic tool was used.

The article "Investigating the Effect of Keyboard Distance on the Posture and 3D Moments of Wrist and Elbow Joints among Males Using OpenSim" was published in 2022. Journal: Appl Bionics Biomech.

Parameters such as minimum, maximum, mean, standard deviation, and ROM of the kinematic and kinetic variables were also calculated. Before the test, the markers were placed on the participant's body, and they were asked to maintain a standard anatomical posture with the torso straight, the arms in a vertical position, and the forearms in a horizontal position (90-degree elbow angle). The information obtained from the position of the markers was used as a static test to scale the model. Scaling the model was completed with an error of less than 2 cm. Inverse kinematic and dynamic calculation methods were used to determine ROM and 3D joint moments.

### 2.3. Visual Analog Scale (VAS)

Participants completed a subjective discomfort assessment for each limb before and immediately after completing the task. This was done by placing a tick mark on a 10 cm continuous visual analog scale [28].

### 2.4. Experimental Conditions

A QWERTY keyboard was randomly placed at three horizontal distances between the monitor and the user on the desk surface (Figure 2). These distances were set up as follows: the edge of the desk (T1), 8 cm away (T2), and 15 cm away (T3) from the edge of the desk. The conditions of the study were the same for all participants. The participants' age and anthropometric variables, including weight, body mass index, elbow, hip, knee, popliteal, eye height, and arm length, were recorded, and workstation dimensions were adjusted according to ANSI/HFES-100-2007 standard for each participant [29]. A 17-inch flat monitor was positioned at eye height and arm length of the participants. The 1/3rd top section of the monitor screen was always adjusted to each participant's eye level. The chair and the desk height were adjusted to individuals' knee height and elbow height, and the keyboard was aligned to the center of their bodies. The mouse was always located on the right side of the keyboard. Environmental conditions were the same in all trials for all participants, and a standard office chair was used.

Figure 3 demonstrates the experimental setup in which participants had to complete writing and reading comprehension for about 10 minutes (2 intervals of 5 minutes). A specific text was provided to the participants to type; the font size and document zoom level in Microsoft word were adjusted, respectively, to 14 and 120%, in all trials. After completing each trial, the participant rested for 5 minutes. The dynamic assessment was performed when participants had to complete the task.

The article "Investigating the Effect of Keyboard Distance on the Posture and 3D Moments of Wrist and Elbow Joints among Males Using OpenSim" was published in 2022. Journal: Appl Bionics Biomech.

Reflective markers were placed, according to the standard protocol described [29], on the participants' 7th cervical vertebrae, acromion process, arm, forearm, sternum, the base of metacarpal 1, 2, and 5, handle, medial-lateral elbow joints, and medial-lateral styloid processes of the wrist on both the right and left sides [30].  Figure 4 shows markers placement for the motion capture system.

### 2.5. Data Analysis

The statistics of mean and standard deviation were used to describe the quantitative variables. The normal distribution of the variables was determined by the Kolmogorov–Smirnov test. The Friedman test was used for comparing the differences between ROM, mean values of the moments, and subjective scores of VAS at the three keyboard distances. The Wilcoxon test was used for two-by-two comparisons at different distances. SPSS (version 16) was used for statistical analysis, and all analyses were performed at a significance level of 0.05.

## 3. Results

The mean participants' age, weight, and height were 27 (2.8) years, 73 (5.6) kg, and 178 (3.9) cm, respectively.

The OpenSim software defined the local coordinate system of joints so that the flexion, radial deviation, and pronation were positive, and extension, ulnar deviation, and supination were negative.  Table 1 shows the mean ROM of flexion-extension and deviation of the right and left wrists.

The Friedman test showed that both wrists' ROM of flexion-extension and ulnar-radial deviation differed significantly at the three different keyboard distances (*P* value < 0.05). Two-by-two comparisons of the right wrist showed a significant difference at all three distances.

In contrast, for the left wrist, only a difference was observed between T1 or T3 and T2 (*P* value < 0.05), and no significant difference was seen between T1 and T3 distances (*P* value > 0.05).  Table 2 shows the mean ROM measured for the left and the right elbows at different keyboard distances. Flexion-extension, supination, and pronation of the elbows are presented in this table.

The Friedman test results showed a significant difference between the elbow flexion and extension at different keyboard distances. Moreover, the right elbow's ROM of supination and pronation at three different keyboard distances showed statistically significant differences (*P* value < 0.05). There were no significant differences between the left elbow supination and pronation at three keyboard distances (*P* value = 0.063).

The Wilcoxon test for two-by-two comparison in elbow flexion and extension showed a significant difference at the T1, T2, and T3 positions. However, in the supination and pronation movements of the right and left elbows, a significant difference was observed only between T1 or T3 and T2 (*P* value < 0.05), and no significant difference was seen between T1 and T3 (*P* value > 0.05).

The article "Investigating the Effect of Keyboard Distance on the Posture and 3D Moments of Wrist and Elbow Joints among Males Using OpenSim" was published in 2022. Journal: Appl Bionics Biomech.

Figure 5 shows the comparison of mean values of the moments of left and right wrist flexion-extension. The results of these variables are presented separately for different keyboard distances. The calculated moments were normalized based on the participant's weight. The Friedman test was used to differentiate distances shown in each figure by comparing different keyboard distances. The mean values of wrist flexion and extension moments were different at the three keyboard distances, but the difference between these values was not statistically significant (*P* value > 0.05).

Figure 6 shows the mean values of the wrist ulnar-radial deviation moments at the three keyboard distances, T1, T2, and T3, respectively. As can be seen, at distances T2 and T3, the values for the right and left hands are equal (0.01 and 0.03 Nm/kg, respectively). Based on the results, the difference among the three distances is not statistically significant (*P* value > 0.05).

Figure 7 shows the mean values of elbow flexion and extension moments at three keyboard distances (Nm/kg). The mean values of elbow flexion and extension are presented separately for different keyboard distances. Despite the difference in the mean values of elbow flexion and extension at three keyboard distances, no significant difference was observed between these values (*P* value > 0.05).

Figure 8 shows the mean values of elbow supination-pronation moments at the three distances of the keyboard. The mean values for the right and left hands are presented separately for different keyboard distances based on the results. The statistical test did not show significant differences among the three keyboard distances (*P* value > 0.05).

Table 3 shows the results of the participants' subjective assessment of discomfort at different keyboard distances after 10 minutes of predefined computer tasks. According to these results, the highest discomfort was reported when the keyboard was at distance T1.

As shown in Table 3, the mean discomfort scores at the three keyboard distances are significantly different for wrists but not for elbows.

## 4. Discussion

The present study was aimed at quantifying the effects of different keyboard positions on the posture and 3D moments of wrist and elbow joints. Accordingly, the participants were asked to perform standard predefined computer tasks in three keyboard positions. The results showed that the keyboard distance affected the posture and the upper extremity joint moments.

The article "Investigating the Effect of Keyboard Distance on the Posture and 3D Moments of Wrist and Elbow Joints among Males Using OpenSim" was published in 2022. Journal: Appl Bionics Biomech.

The highest wrist flexion and radial deviation occurred at T1, and with increasing the distance of the keyboard from the body, these values decreased. The lowest flexion and radial deviation occurred at T2. In this study, wrist flexion decreased by increasing the keyboard distance to 8 cm (T2). This is similar to the results of the study carried out by Kotani et al., in which by increasing the distance, the wrist flexion decreased [16].

In our study, the radial deviation decreased to near the neutral posture by increasing the distance of the keyboard from the body, as reported by Cook et al. [12]. It can be concluded that at T2, the risk of MSDs in wrists and elbows is lower than at the other two distances.

By increasing the keyboard distance from T1 to T2, the ROM of left wrist flexion decreased about 95% (*P* value < 0.05). In general, the ROM of left wrist flexion decreased as the distance increased (from T1 to T2 and T3), similar to the results of Kotani et al.

When the position of the keyboard changed from T1 to T2, the ROM of the left wrist radial deviation decreased significantly (*P* value < 0.05), similar to the results of Kotani et al. However, at distance T3, this value slightly increased compared to distance T1 (*P* value > 0.05), which was not in agreement with the results of Kotani et al. [16]. In the right wrist, an average of 83% in flexion and 89% in ulnar-radial deviation values reduction was observed at T2 than two positions.

By increasing the distance to T2, the left wrist flexion and radial deviation decreased significantly an average about 93% (*P* value < 0.05). This was consistent with the results of previous studies [12, 16]. However, at T3, the radial deviation increased. This part of our results was not similar to those of Ketone et al. [16]. The study by Lindberg et al. and Qing et al. showed that wrist flexion and extension, even in a short time, can lead to wrist MSDs in prolonged working time [31, 32]. As the keyboard distance increased, the ROM decreased, and the lowest value occurred at T2. At the other two distances, the ROM increased.

According to the study carried out by Waersted et al., elbow extension and flexion could contribute to elbow MSDs [3]. The ROM in flexion-extension, supination, and pronation of the right elbow at the three keyboard distances revealed a significant difference (*P* value < 0.05). An average of 95% flexion and 76% supination-pronation values reduction was observed at T2 than two positions. In the left elbow, the ROM of flexion-extension showed an average 85% reduction at the three keyboard distances (*P* value < 0.05). Supination and pronation decreased by increasing the distance of the keyboard from T1 to T2 and form T3 to T2. Still, no significant difference was observed (*P* value > 0.05), which was similar to the results of the studies by Marcus et al., Kotani et al., and Cook et al. [10, 12, 16]. This can be explained by the fact that all participants were right-handed, and the left arm was passive [33].

The article "Investigating the Effect of Keyboard Distance on the Posture and 3D Moments of Wrist and Elbow Joints among Males Using OpenSim" was published in 2022. Journal: Appl Bionics Biomech.

There are differences in the wrist and elbow kinematics at the three distances, as shown in Tables 1 and 2. These differences might be due to the fact that when the keyboard was moved away from the edge of the desk, the subjects placed their distal forearms on the desk to support their upper arms and shoulders, so wrist flexion, radial deviation, and pronation decreased. When the keyboard was moved further away, the proximal forearms and the elbows were placed on the desk to support the upper arms and shoulders, so wrist extension, ulnar deviation, and supination increased [12].

The subjective assessment of discomfort showed that when the keyboard was placed on the edge of the desk, the wrists were mostly discomfort, which seemed to be due to excessive flexion of the wrists at this distance. The results of this assessment are similar to those of Marcus et al. [10].

The changes were more significant in kinematic than in kinetic variables. Therefore, the wrist and elbow moments did not show a statistically significant difference at the three distances of the keyboard. This is because the active muscles are fixed (static activity) during computer tasks. In other words, by changing the horizontal distance of the keyboard from the edge of the desk, the working muscles have static activity at the beginning and end of the task cycle. The moments at T1 and T3 setups are very close to each other but these ROM values are different; these differences might be because at start motion the joint angles were away from neutral position. In fact, in our study, ROM reported that shows a range of joint motions.

The changes in the angles of the joints, no matter how small, affect the muscles. For more changes in the angles of the joints and for a longer duration of joint involvement, the muscles are more involved, and the risk of injuries increases. This is because no muscles were deactivated, but they acted as constant mover or stabilizer. The results of this part are similar to those of the study by Kotani et al. [16].

In this study, the OpenSim software was used to evaluate the joint moments in three dimensions (3D) for making it possible to calculate the moments around the coordinate axes *x*, *y*, and *z*. This study had some limitations, such as testing only right-handed male participants in the age range of 25-30 years and not considering other workstation elements, e.g., monitor, desk, and chair. Moreover, due to the short duration of the tests, the results may differ in studies with more extended test duration. These limitations should be considered in future studies.

The article "Investigating the Effect of Keyboard Distance on the Posture and 3D Moments of Wrist and Elbow Joints among Males Using OpenSim" was published in 2022. Journal: Appl Bionics Biomech.

## 5. Conclusion

According to the results of this study, changes in the horizontal distance of the keyboard can affect the upper extremity kinematics and moments. The keyboard distance has a significant impact on the posture of the upper limbs. However, when the joints are close to their neutral position, the risk of MSDs decreases. In general, when the keyboard is placed on the edge of the desk, it is expected that the flexion, radial deviation, and pronation are at high levels, as the most likely cause of the disorders. By increasing the keyboard distance to 8 cm from the edge of the desk, the values of these variables decrease significantly. However, increasing the distance to 15 cm slightly increases these values.

Accordingly, appropriate postures of wrists and elbows can be maintained when the keyboard is at a distance of 8 cm from the edge of the desk. This reduces the risk of MSDs in the upper extremities. Therefore, based on the results of this study, the keyboard distance should be neither on the edge of the desk nor at a large distance from the individual's body. Further studies on various other distances conducted on male and female participants can provide more detailed information.

## Figures and Tables

**Figure 1:** Anterior (a) and lateral (b) view of OpenSim upper limb model.

**Figure 2:** The three distances of the keyboard. T1: keyboard positioned at the edge of the desk, T2: 8 cm away from the edge of the desk, and T3: keyboard positioned at 15 cm away from the edge of the desk.

**Figure 3:** Experimental setup in the motion capture laboratory. (a) Right and (b) left view.

**Figure 4:** Placement of markers for optical motion capture system. (a) Anterior, (b) posterior, and (c) lateral view.

**Figure 5:** Mean values of flexion-extension of the wrists moments in three distances of the keyboard (Nm/kg).

**Figure 6:** Mean values of ulnar-radial deviation of the wrists moments in three distances of the keyboard (Nm/kg).

**Figure 7:** Mean values of flexion-extension of the elbows moments in three distances of the keyboard (Nm/kg).

**Figure 8:** Mean values of supination-pronation of the elbows moments in three distances of the keyboard (Nm/kg).

**Table 1:** Mean ROM ± SD value of flexion-extension and deviation of the wrists in three distances of the keyboard (°).

Variable		Keyboard distances			*P* value^∗^
		T1	T2	T3	
Right wrist	Flexion-extension (°)	24.51 ± 18.51	2.96 ± 1.03	14.86 ± 9.15	**0.012**
	Ulnar-radial deviation (°)	18.61 ± 14.74	1.46 ± 0.74	11.32 ± 9.74	**0.041**
Left wrist	Flexion-extension (°)	22.61 ± 17.74	1.12 ± 0.12	17.55 ± 11.04	**0.026**
	Ulnar-radial deviation (°)	18.57 ± 13.23	1.13 ± 0.01	19.14 ± 16.02	**0.035**

^∗^Friedman test. Bolded values indicate statistically significant results. T1: trial 1; T2: trial 2; T3: trial 3.

The article "Investigating the Effect of Keyboard Distance on the Posture and 3D Moments of Wrist and Elbow Joints among Males Using OpenSim" was published in 2022. Journal: Appl Bionics Biomech.

**Table 2:** Mean ROM ± SD values of the elbow flexion-extension and pronation-supination in three distances of the keyboard (°).

Variable		Keyboard distances			*P* value^∗^
		T1	T2	T3	
Right elbow	Flexion-extension (°)	26.00 ± 18.49	0.99 ± 0.01	17.42 ± 11.29	**0.001**
	Pronation-supination (°)	13.00 ± 8.87	2.40 ± 0.94	8.84 ± 6.02	**0.043**
Left elbow	Flexion-extension (°)	10.31 ± 7.79	1.15 ± 0.18	6.85 ± 2.93	**0.039**
	Pronation-supination (°)	11.06 ± 5.92	3.01 ± 0.82	8.30 ± 3.01	0.063

^∗^Friedman test. Bolded values indicate statistically significant results. T1: trial 1; T2: trial 2; T3: trial 3.

**Table 3:** Mean (standard deviation) scores of subjective discomfort assessment (*n* = 12).

Region	T1	T2	T3	*P* value^∗^
Right wrist	3.12 (0.23)	2.01 (0.41)	1.27 (0.15)	**0.012**
Left wrist	2.96 (0.8)	1.88 (0.3)	1.49 (0.2)	**0.037**
Right elbow	2.78 (0.12)	2.16 (0.41)	1.93 (0.33)	0.962
Left elbow	1.76 (0.04)	1.48 (0.08)	1.23 (0.13)	0.124

^∗^Friedman test. Bolded values indicate statistically significant results. Zero meant no discomfort, and 10 represented the highest discomfort.

## Data Availability

The processed data are available from the corresponding author upon request.
